The article "Auxiliary Pneumonia Classification Algorithm Based on Pruning Compression" was published in 2022. Journal: Comput Math Methods Med.

# Auxiliary Pneumonia Classification Algorithm Based on Pruning Compression

**DOI:** 10.1155/2022/8415187

**Published:** 2022-07-18

**Authors:** Chao-Peng Yang, Jian-Qing Zhu, Tan Yan, Qiu-Ling Su, Li-Xin Zheng

**Affiliations:** ^1^College of Engineering, Huaqiao University, Quanzhou 362021, China; ^2^The 910th Hospital of the Joint Support Force of the Chinese People's Liberation Army, Quanzhou 362008, China

## Abstract

Pneumonia infection is the leading cause of death in young children. The commonly used pneumonia detection method is that doctors diagnose through chest X-ray, and external factors easily interfere with the results. Assisting doctors in diagnosing pneumonia in patients based on deep learning methods can effectively eliminate similar problems. However, the complex network structure and redundant parameters of deep neural networks and the limited storage and computing resources of clinical medical hardware devices make it difficult for this method to use widely in clinical practice. Therefore, this paper studies a lightweight pneumonia classification network, CPGResNet50 (ResNet50 with custom channel pruning and ghost methods), based on ResNet50 pruning and compression to better meet the application requirements of clinical pneumonia auxiliary diagnosis with high precision and low memory. First, based on the hierarchical channel pruning method, the channel after the convolutional layer in the bottleneck part of the backbone network layer is used as the pruning object, and the pruning operation is performed after its normalization to obtain a network model with a high compression ratio. Second, the pruned convolutional layers are decomposed into original convolutions and cheap convolutions using the optimized convolution method. The feature maps generated by the two convolution parts are combined as the input to the next convolutional layer. Further, we conducted many experiments using pneumonia X-ray medical image data. The results show that the proposed method reduces the number of parameters of the ResNet50 network model from 23.7 M to 3.455 M when the pruning rate is 90%, a reduction is more than 85%, FIOPs dropped from 4.12G to 523.09 M, and the speed increased by more than 85%. The model training accuracy error remained within 1%. Therefore, the proposed method has a good performance in the auxiliary diagnosis of pneumonia and obtained good experimental results.

## 1. Introduction

Pneumonia is one of the most common infectious diseases in clinical medicine. It has a short onset cycle and a complex etiology [1]. Children and the elderly with relatively low immunity are especially susceptible. According to the World Health Organization, in 2016 alone, more than 800,000 people died of pneumonia worldwide, more than malaria, AIDS, and measles combined [2]. Therefore, pneumonia must be diagnosed and treated promptly. Clinical diagnosis of lung diseases mainly relies on radiologists to observe X-ray images as a reference [3]. At the same time, X-ray has the advantages of fast imaging speed, low cost, and moderate imaging quality, making it widely used in clinical practice. The daily diagnosis of pneumonia requires a high level of expertise and clinical experience [4]. More importantly, it is inevitable that doctors suffer from visual fatigue, misdiagnosis, and missed diagnoses during the diagnostic process. Therefore, it is hugely challenging for doctors to spend much time every day observing a large number of lung images and accurately diagnosing the symptoms of pneumonia. The average image and the pneumonia image are shown in Figure 1.

The article "Auxiliary Pneumonia Classification Algorithm Based on Pruning Compression" was published in 2022. Journal: Comput Math Methods Med.

Medical image classification is one of the hot research areas in computer vision [5]. With the rapid development of convolutional neural network (CNN), many researchers have introduced it into the medical industry and are widely used in medical imaging [6, 7]. Scholars have carried out research at home and abroad on chest X-ray images. In the auxiliary diagnosis of pneumonia, domestic and foreign scholars have proposed their methods [8]. However, due to the lack of memory and computing power of the current ordinary PC equipment, large network models such as Inception, DenseNet121, and ResNet50 cannot be effectively deployed, resulting in the inability to be widely and effectively used in clinical medicine.

In response to the large-scale network models, a series of methods have been proposed to study compact deep neural networks, such as network pruning [9], low-bit quantization [10], and knowledge distillation [11, 12]. Among them, network pruning is an effective method for compressing large network models so that the model can better balance the inference speed and model accuracy. In network pruning, the channel pruning method, which uses the channel between the network layers to prune, can ensure the structural integrity of the original model and at the same time have a higher compression ratio, so it has been widely studied. The channel pruning method mainly uses the channels from the BN layer to the convolution layer (or neurons in the fully connected layer) to filter and prunes the unnecessary channels, to achieve the effect of model compression. It has been widely studied because this method does not destroy the original model structure and has a better compression effect.

In view of the application requirements of simple, high-precision, and small-memory aided diagnosis methods for pneumonia, we propose a custom layer channel pruning (CP) method, which uses the channel weights of each layer in the network model to sort and further identify and delete the associations among them. Expressly, we set a separate pruning number for each layer to better control the pruning range. At the same time, it also guarantees a different number of prunings required for specific layer channels in ResNet50 [13]. Then, the cheap convolution method [14] is combined with channel pruning to designing the CPGResNet50 structure. The pruned convolution layer is mainly decomposed into two parts: the original convolution part and the cheap convolution part. Among them, half of the feature channels of the original convolution layer are intrinsic feature maps, while the other half of the feature channels are generated by simple linear operations. Experiments show that this method achieves better performance in overall model parameters and computational complexity.

The article "Auxiliary Pneumonia Classification Algorithm Based on Pruning Compression" was published in 2022. Journal: Comput Math Methods Med.

## 2. Related Work

This section reviews current CNN-based pneumonia-aided diagnosis methods, as well as current methods for mitigating neural networks. We divided the analysis into two parts the deep learning-based pneumonia-assisted classification method and the model compression method design.

### 2.1. Auxiliary Classification of Pneumonia

Compared with traditional simple learning, the difference between deep learning is that the former can “autonomously” learn through a multilayer nonlinear structure to characterize data characteristics. Computer-aided diagnosis systems have been gradually introduced into clinical practice with the development of computer and digital image processing technology. Chinese and foreign scholars have proposed many different methods for automatically identifying pneumonia images. According to the characteristics of pneumonia images, in 2020, Qi et al. [12] used the characteristics of medical images to pretrain the InceptionV3 model with a deeper and more complex structure through the method of knowledge distillation and put the well-trained “knowledge” (practical information) to the AlexNet [15] model. However, the number of parameters of the AlexNet model itself has reached 60 million, which also has specific requirements for hardware. In 2018, Rajpurkar et al. [16] proposed a 121-layer convolutional neural network, trained on 112,120 labeled lung X-ray image datasets ChestX-ray14, and detected 14 different lung diseases. During the process, 11 achieved similar or better performance to radiologists. In 2020, Gabruseva et al. [17] used SE-ResNext101 [18] as the base model with ResNext as the backbone network and achieved second place in the Kaggle Pneumonia Region Detection Challenge with the following modifications. The layers of the two types of pneumonia classification models both exceed 100 layers, and their classification speed and parameter amount pose significant challenges to their clinical applications.

The article "Auxiliary Pneumonia Classification Algorithm Based on Pruning Compression" was published in 2022. Journal: Comput Math Methods Med.

### 2.2. Design of Model Compression Method

Given many parameters, extended training and fitting time, and high hardware requirements of current network models, researchers have proposed different methods, such as compact model design, knowledge distillation, quantization, and model pruning.

#### 2.2.1. Compact Models

A series of efficient network architectures have gained popularity due to their compact size and low computational requirements, including MobileNets [19] and ShuffleNetV2 [20]. MobileNets are a family of lightweight deep neural networks based on depthwise separable convolutions. MobileNetV2 [21] proposes a reverse residual block, and MobileNetV3 [22] further leverages AutoML techniques [23] to achieve better performance with fewer floating-point numbers. ShuffleNet [24] introduced a channel shuffling operation to improve the exchange of information flow between channel groups. ShuffleNetV2 [20] further considers actual speed on target hardware for compact design. Although these models have achieved good performance with little failure probability, they may not provide good generalization performance for chest pneumonia recognition requiring shallow texture features and in-depth feature information. Therefore, the above compact model is not well suited for the classification of lung X-ray images.

#### 2.2.2. Quantization

The parameters are stored as 32-bit floating-point numbers in CNN, which can effectively reduce the size of training CNN by reducing the number of bits of weights and activation parameters. In quantization, weights are represented by reducing the number of bits required to store each weight per weight. This idea can also be extended further to represent gradients and activations in quantized form. Weights can be quantized to 16-bit, 8-bit, and 4-bit or even 1-bit (this is a particular case of quantization, where binary values, called weight binarization, only represent weights) [25].

#### 2.2.3. Knowledge Distillation

The knowledge learned by a more extensive bulky network (teacher model) trained on a large dataset is transferred to a smaller and lighter network, called a student model, which can generalize well-unseen data. Qi et al. [12] used AlexNet and InceptionV3 to obtain better results with the knowledge distillation method to classify pneumonia. Although its accuracy has been improved to a certain extent, its accuracy is still lacking for clinical medical needs.

The article "Auxiliary Pneumonia Classification Algorithm Based on Pruning Compression" was published in 2022. Journal: Comput Math Methods Med.

#### 2.2.4. Model Pruning

In CNNs, many parameters are redundant, and these parameters do not contribute much during training, which reduces the error and generalizes the network. Therefore, some parameters that have little effect on the network can be discarded after training. The primary purpose of pruning is to reduce the storage requirements of the model and make it storage-friendly. By pruning the parameters/filters of the convolutional layers, the amount of computation can be reduced, and the inference process can be accelerated. In a CNN model, different connections have different degrees of importance. Therefore, eliminating less impactful connections can significantly reduce CNN models' storage, computational cost, energy, and inference time. According to the granularity of pruning, pruning can be divided into structured pruning and unstructured pruning. Among them, unstructured pruning has finer granularity and can prune any parameters without limit, such as weight pruning [26, 27]. Such methods also destroy the model structure and cannot effectively speed up [28]. Structured pruning [29] has a coarser granularity and uses different weights of filters or feature maps to prune and delete certain filters or channels. In 2018, Mocanu et al. [30] used the L1-norm on the filter to select unimportant filters for deletion. In 2019, Molchanov et al. [31] used sparse regularization and low-loss filters for removal. Channel pruning is similar to filter pruning in that it removes redundant parts of the model structure. Among them, channel pruning removes the entire redundant filter, so that similar ResNet and DenseNet have multibranched network structure dimension matching. In 2016, Song et al. [32] proposed multiple compression stages, using each step of the compression operation separately, ignoring the interaction between different compression operations. Dubey et al. [33] first used filter pruning to compress the weights and then decomposed the weights based on the coreset decomposition method.

Other tailoring methods have varying degrees of application requirements that are not suitable for pneumonia diagnosis and cannot meet our experimental requirements. First, the pruning scale setting is limited by the channel pruning method. Due to the different number of channels between the layers of the network model, when the channel pruning rate reaches a specific size, it may cause all channels of some layers to be pruned, resulting in the model being unable to work. Second, taking the method of Liu et al. [34] as an example, its network thinning method uses sparseness to make the weight gap between channels larger and requires sparse training first, which increases the complexity of the experiment. Although the weight-level sparse cropping can produce a more significant compression rate, it requires specific hardware and libraries to achieve a performance improvement, which cannot meet our requirements. The layer-level sparse clipping requires clipping of the complete layer, which makes it less flexible. Moreover, in the actual experiment, removing the layer only when the number of network layers reaches more than 50 layers can obtain better results while ensuring accuracy. Layer channel pruning is a compromise between the above two methods. It has vital flexibility and will not be limited by the model structure. At the same time, the algorithm integrates and optimizes the convolution, which effectively avoids the collapse of the accuracy caused by the extreme pruning rate of the model.

The article "Auxiliary Pneumonia Classification Algorithm Based on Pruning Compression" was published in 2022. Journal: Comput Math Methods Med.

Our contributions are summarized as follows:

1. A channel pruning decomposition method is proposed. We design controllable hierarchical channel pruning and process the original classification network model in combination with the optimized convolution operation so that the network model achieves the effect of balancing accuracy and speed in the pneumonia classification experiment
2. Using the deep learning method of channel pruning and decomposition to research pneumonia medical images can obtain higher accuracy in classifying pneumonia medical X-ray image data. At the same time, the computational cost can be significantly saved

## 3. Method

In this section, we will divide into three parts. First, we use the BasicBlock of ResNet50 as the unit to prune the three-layer convolutional layer channel. Then by analogy to the whole model, CPResNet50 with custom channel pruning is designed. Then further, the method of decomposing convolution is designed to design GResNet50 for the convolutional layer operations that occupy the main computational load of the model, and its performance is further evaluated. Finally, channel pruning and optimized convolution are fused to compress the model further to design CPGResNet50.

### 3.1. Self-Regulating Channel Pruning

The Method of CPResNet50: In the neural network model structure, many convolutional layers are usually included, and the convolutional operation of the convolutional layer will generate a large amount of computational cost. As a structured pruning method, channel pruning uses different weights of feature map channels to distinguish and prune channels with lower weights, thereby reducing the input of convolutional layers and reducing computational resources.  Figure 2 shows the operation of the pruning block. The left side is one of the BasicBlock blocks of ResNet50, and the right side is the pruned BasicBlock block.

The article "Auxiliary Pneumonia Classification Algorithm Based on Pruning Compression" was published in 2022. Journal: Comput Math Methods Med.

The network thinning method proposed by Liu et al. [34] in 2017 used the feature channel to be cropped by introducing a scaling factor *λ* in the BN layer. The specific method is that the feature channel generated after the convolution layer uses the shrink factor *λ* as the main judgment parameter in the batch normalized BN layer; that is, when the shrink factor *λ* is smaller, the corresponding channel less critical is cropped. By pruning the unimportant channels of each layer, the overall compression of the model is achieved at one time. During training, *L*_1_ regularization is added to the scale factor of the BN layer to achieve the effect of sparseness so that the unimportant channels can be identified by the scale factor of the BN layer approaching 0, formulated as

(1) $$\begin{array}{c} L=\underset{\left(x,y\right)}{\sum }l\left(f\left(x,W\right),y\right)+\gamma \underset{\gamma \in \Gamma }{\sum }g\left(\lambda \right), \end{array}$$

where *λ* represents the scale factor, *λ* stands for the penalty sparsity, *g*(*λ*) = |*λ*| is the penalty on the scale factor, (*x*, *y*) denote the training input and target, and*W*is obtained at the trainable weight. Inspired by Liu et al. [34], we propose a new method for pruning convolutional channels individually for each layer. First, the parameters and number of channels of each BN layer are obtained, and the BN layer performs the following transformations:

(2) $$\begin{array}{c} y_{i}^{\left(b\right)}=BN{\left(x_{i}\right)}^{\left(b\right)}=\lambda \cdot \left(\frac{x_{i}^{\left(b\right)}-\mu \left(x_{i}\right)}{\sqrt{\sigma {\left(x_{i}\right)}^{2}+\varepsilon }}\right)+\beta , \end{array}$$

where *x*_*i*_^(*b*)^ represents the value of the *i*-th input node of the layer when the *b*-th sample of the current batch is input, *x*_*i*_ is the row vector composed of [*x*_(1)*i*_, *x*_(2)*i*_, ⋯, *x*_(*m*)*i*_], the length is the batch size *m*, *μ* and *σ* are the mean and standard deviation of the row,*ε*, to prevent the extremely small (negligible) amount introduced by division by zero, and *λ* and *β* are the scale and shift parameters of the row.

Then, directly sort the channel weights of the normalization layers of the first two convolutional layers of each bottleneck block of ResNet50 from small to large, and finally, prune the features of each layer according to the number of channels of the original convolutional layers of each layer. The most significant advantage of this is that there is no need to introduce a scale factor for sparse training of the overall model, which will not cause additional computational overhead to the network. Among them, only the two convolutional layers of the bottleneck block are pruned, mainly to avoid the short-circuit connection at the Bottleneck in the ResNet50 module and ensure the integrity of the overall structure model to ensure the connection between blocks. In practice, *C*_out_ is the number of output channels of the convolution layer, *C*_in_ is the number of input channels of the convolution layer, *K*_*h*_ and *K*_*w*_ are the convolution kernel height and width of the convolution layer, respectively, and *λ* is the pruning ratio of the convolution layer. Then, the parameters of this layer are

(3) $$\begin{array}{c} P_{i}=\left(K_{h}\cdot K_{W}\cdot C_{\text{in}i}\right)\cdot \left(C_{\text{out}i}-C_{\text{out}i}\cdot \lambda_{i}\right)+\left(C_{\text{out}i}-C_{\text{out}i}\cdot \lambda_{i}\right), \end{array}$$

where *i* represents the convolution of the *i*-th layer and *P*_*i*_ represents the number of parameters generated by the *i*-th layer. According to the above formula, the parameter amount of the layer *i* will be reduced *λ*_*i*_ according to the pruning ratio of this layer. The unimportant feature channels are removed through the above operations, while the vital feature channels are retained. The specific operation is shown in Figure 3.

The article "Auxiliary Pneumonia Classification Algorithm Based on Pruning Compression" was published in 2022. Journal: Comput Math Methods Med.

Using the controllable layer channel pruning method, the pruning rate of each convolutional layer channel can be designed so it has a high degree of flexibility. At the same time, because the channels between convolutional layers are used for pruning, this method can even achieve single-channel (the number of channels between convolutional layers is 1) pruning, which can achieve an excellent model compression ratio.

### 3.2. Decomposed Convolution after Pruning

During channel pruning, as the number of channels between each layer is fixed, this can lead to a concentration of model training on localized areas in the later pruning stages. The consequence is that an overall analysis is not possible, making the model lack generalization. Drawing on the cheap convolution module of Ghost [14], it solves the above problems to a certain extent and further compresses the model based on channel pruning. First, the decomposed convolution operation is performed on the pruned model to obtain the recompression of the model scale. The specific operation is that in a convolution operation containing *n* feature channels in a particular layer, *m* (*m* < *n*) channels are obtained by linear operation. At the same time, ensure that the filter size, stride, padding, and other hyperparameters in linearly generating features are the same as those in ordinary convolution (Formula (4)) to keep the spatial size of the output feature map (i.e., *h*_0_and *w*_0_) consistent. The actual convolution operation is as follows:

(4) $$\begin{array}{c} Y=X\times f+b, \end{array}$$

where *Y* represents the output after convolution, is the input of the convolution, *f* is the filter, and *b* is the offset.

The article "Auxiliary Pneumonia Classification Algorithm Based on Pruning Compression" was published in 2022. Journal: Comput Math Methods Med.

Cheap convolution is

(5) $$\begin{array}{c} Y^{\prime }=X\times f^{\prime }, \end{array}$$

where represents the output after convolution and *f*′ is the filter. In order to reduce the computational complexity, the *b* bias is set to 0 here.

To further obtain the required *n* feature maps, a series of cheap linear operations are performed on each intrinsic feature in *y*_0_ to generate s cheap features according to the following function:

(6) $$\begin{array}{c} y_{i,j}=\Phi_{i,j}\left(y_{i}^{\prime }\right),\;\forall_{i}=1,\cdots ,s, \end{array}$$

where *y*_*i*,*j*_ is the -th eigenfeature map of *y*. *Φ*_*i*,*j*_ in the above function is the *j*-th linear operation to generate the *j*-th cheap feature maps (except the last one); that is, *y*_*i*_′ can have one or more cheap feature maps {*y*_*i*,*j*_}_*j*=1_^*s*^. Using Equation (6), the feature map *n* = *m* × *s* of *Y* = [*Y*_1_, *Y*_2_, ⋯, *Y*_*ms*_] can be obtained as the output data of the Ghost module.  Figure 4 shows the details of the convolution decomposition structure diagram.

The specific parameter calculation formula is as

(7) $$\begin{array}{c} P_{i}=\left(K_{h}\cdot K_{W}\cdot C_{\text{in}i}\right)\cdot \frac{p_{\text{out}i}\cdot \left(n-s\right)}{n}+p_{\text{out}i}\cdot \left(1+\frac{s}{n}\right), \end{array}$$

where *p*_out*i*_ = *C*_out*i*_ − *C*_out*i*_ · *λ*_*i*_ is the number of output channels of the *i*-th layer after the channel, *s* is the number of cheap feature maps, and *n* is the total number of output features after pruning this convolutional layer.

### 3.3. Decomposed Convolution after Pruning

In the pruning method, with the further increase of the pruning degree, the loss to the model is also more significant, which leads to the collapse of the training accuracy. Ghost's method of optimizing convolution can make up for this problem to a certain extent. When the pruning rate is more likely to cause the accuracy to collapse, the optimized convolution method is used to compress the model scale further while preventing the progress from collapsing.

The specific structure and operation of the method are shown in Figure 5, which mainly depicts the most critical convolutional layer. The structure of ResNet50 includes a convolution layer at the beginning and a maximum pooling layer and 16 convolution blocks of BasicBlock in the middle. Each convolution block contains three layers of convolution layers. The shortcut is ignored here, and the end is mainly composed of the average pooling layer and a fully connected layer. Figure 5(b) describes the specific process of channel pruning and fusion optimizing convolution, including the size or dimension of each layer output. Since ResNet has a shortcut structure, to ensure the dimensional consistency of the bottleneck structure of the model, pruning will be applied to the first and second-layer convolutional structure in BasicBlock.

The article "Auxiliary Pneumonia Classification Algorithm Based on Pruning Compression" was published in 2022. Journal: Comput Math Methods Med.

Our study uses channel pruning first, followed by optimized convolution operations. In theory, if the convolution operation is performed first, the original convolution layer becomes the original convolution layer and the cheap convolution layer (where the cheap convolution selects the best 50% ratio for the model). The number of channels of the original convolutional layer and the cheap convolutional layer becomes half of the number of channels when the convolutional layer is input. Then, channel pruning is performed on the model since the number of channels is reduced by half and the number of pruning layers is doubled; channel pruning is not used. Under the same pruning rate, optimizing the pruning before convolution and optimizing the pruning after convolution, the number of remaining channels in each layer of the former will be much larger than that of the latter. The model integrity is better, and it is easier to obtain higher accuracy.

## 4. Experiments

In this section, we first train on the pneumonia dataset with the proposed CPResNet50 to verify its effectiveness. Then, using the decomposed convolutional CPGResNet50 network will further test the effect on pneumonia image classification.

1. Datasets and settings: the dataset used in this paper is ChestX-ray2017, a public dataset based on the X-ray scan database of pediatric patients aged 1 to 5 years in Guangzhou Women and Children's Medical Center [35]. The ChestX-ray2017 dataset contains 5856 chest X-ray images in JPEG, collected and labeled from children. X-ray medical images from 5232 patients include 4273 pneumonia images and 1583 typical images. Among them, there are 4169 training images and 1687 test images. Common data preprocessing strategies such as random cropping and flipping are adopted during training.
2. Evaluation indicators: the evaluation methods we used in the experiment are as follows: confusion matrix, accuracy rate (Acc), recall rate, model parameter quantity, model Flops, memory usage, and MAdd (addition and multiplication operation). The confusion matrix, also known as the error matrix, can be used as an intuitive representation of the model classification effect. Furthermore, through the analysis of confusing evidence, it can be concluded which type of model training is more difficult to classify, such as whether the disease is accurate. Among them, the precision rate and recall rate are used to analyze the model's accuracy in predicting pneumonia results. Model parameters, Flops, memory usage, and MAdd are indicators used to represent the model's size.
3. Experimental setup: to ensure the validity of the experimental data, the same parameters and equipment were used for all experiments. Each time with different pruning conditions and in the comparative experiment, the training is performed 5 times, and the average of the results is taken. The training period is 190; the number of batches is 32; the initial value of the loss rate is 0.1; SGD optimizes all.

The article "Auxiliary Pneumonia Classification Algorithm Based on Pruning Compression" was published in 2022. Journal: Comput Math Methods Med.

### 4.1. CPResNet50 Implementation Details

Use comparative experiments to show the effect of pruning. In order to further demonstrate the effect of CPResNet50 in the field of pneumonia classification, we conducted a large number of experiments for comparative analysis. In order to demonstrate the effectiveness of the method, the experiments will use the training accuracy, model parameters, and FLOPs data as the basis for evaluation and comparison. The experiment first shows the effect of the pruning method. We will use different channel pruning methods to compare the accuracy, parameter quantity, and training speed of the original ResNet50 without the intervention of other factors and network slimming [34], CPResNet50. The training effect under different pruning rates. The specific experimental data are shown in Table 1.

According to the training results of network slimming, CPResNet50 and original ResNet50in the brackets representing the pruning rate, 'normal' represent the model training result without pruning, SResNet50 is the regular training with sparse regularization, and CPResNet50 represents the custom channel pruning training result. In column 4, 10% pruned represents a fine-tuned model that pruned 10% of the channels in the trained model. The trim ratios for parameters and FLOPs are also shown in columns 3 and 5. In the experiment, after the pruning rate of SResNet50 exceeds 70%, all channels in some layers are deleted. Therefore, the pruning rate in the experimental data of SResNet50 does not exceed 70%. According to the experimental data, proper pruning can improve the model's progress compared with the original model. The most considerable improvement is that CPResNet50 achieves a 0.362% improvement compared to the original model at a pruning rate of 50%. At the same time, the accuracy of CPResNet50 is partially improved under the condition of a 90% pruning rate, and the improvement effect is within 0.1%. However, its parameters are compressed by 83.46%, and the training speed is increased by 83.11%, obtaining the best effect.

The article "Auxiliary Pneumonia Classification Algorithm Based on Pruning Compression" was published in 2022. Journal: Comput Math Methods Med.

At the same time, in order to further demonstrate the advantages of the CPResNet50 method, it is compared with VGG16 [36], DenseNet121 [37], GoogLeNet [38], and Inception_v3 in the pneumonia dataset. The experiments mainly compare model classification accuracy, model parameters, training speed (shown in terms of model complexity or FLOPs), and memory usage.

According to Table 2, although GoogLeNet showed the best accuracy in training, when the pruning rate in the CPResNet50 method is 50%, 70%, and 90%, compared with the VGG16, DenseNet121, GoogLeNet, Inception_v3 models, its parameters performance, training speed, and memory footprint.

### 4.2. CPGResNet50 Implementation Details and Results

In CPG experiments, we mainly compare model accuracy and scale. Based on ResNet50, the experiment uses CPG method, SP method, and CP method, respectively. The line chart of accuracy and Flops is shown in Figure 6.

From the ACC and Flops line chart, our method can effectively compress the model to improve the model training speed with little loss of accuracy. Among them, the accuracy error of CPG, SP, and CP is kept within 1%. Flops is that the CPG method is superior to both SP and CP.

To further verify the superiority of CPGResNet50, we compare it with CPResNet50 while we still keep the original training settings. The training results are shown in Table 3.

It can be seen from Table 3 that under the same pruning rate, the model parameters and operation speed are further improved to a certain extent after combining with Ghost's cheap convolution method, and the accuracy loss is always kept within 1.5%. In addition, the reduction of model parameters and the improvement of speed decrease with the increase in pruning rate. When the pruning rate of the model is 90%, the parameter amount can still be reduced by about two percentage points.

In order to further test the compression of the model by the CPResNet50 method, the parameters and model training speed of CPResNet50 are compared with the currently popular lightweight networks MobileNet_V2 and ShuffleNetV2. The comparison results are shown in Table 4.

It can be seen from Table 4 that when the maximum compression rate of 90% is obtained by the CPGResNet50 method, compared with the lightweight models MobileNetV2 and ShuffleNetV2, there is still a particular gap in the number of parameters and Flops, but the gap is not very obvious. When the pruning reaches 90% in the CPGResNet50 method, the parameter amount is only 3.455 M, and the difference between MobileNetV2 is only 1.229 M. Therefore, in the classification of X-ray pneumonia data, CPGResNet50 enables ResNet50 to approach the scale of lightweight models to a certain extent while still having the training accuracy of ResNet50.

The article "Auxiliary Pneumonia Classification Algorithm Based on Pruning Compression" was published in 2022. Journal: Comput Math Methods Med.

## 5. Conclusion and Outlook

To better use the deep learning method for the current clinical pneumonia auxiliary diagnosis, this paper proposes an improved ResNet50 network based on CPResNet50, effectively balancing accuracy and computational requirements and better meeting the clinical pneumonia auxiliary diagnosis needs. The improved method is mainly divided into two parts. The first part is the controllable channel pruning part. This part uses the number of channels in each convolutional model layer to perform layer-by-layer pruning. The pruning rate can be arbitrarily set at the model channel. Achieve the effect of highly compressed models. However, in order to balance the model training accuracy and model training speed, each layer with the best results is selected for channel pruning with a pruning rate of 90% to obtain the best results. The second part is to convert the pruned model. In the convolutional layer, Ghost convolution is used to convert partial convolution operations into linear operations that can save computation. It can ensure that the model achieves maximum compression-optimized performance while maintaining comparable clinical pneumonia additional diagnostic accuracy requirements. Finally, the improved CPGResNet50 model structure is close to the performance of the lightweight network MobileNetV2 in terms of parameters and FLOPs. At the same time, the model achieves better results when training on pneumonia X-ray images. At the same time, there are still some areas for improvement in the method. Pruning can further attempt to screen network layers for more relevant feature information independently. In the later work, we will consider setting an evaluation index of accuracy and model scale and set different pruning rates for channels between different layers. At the same time, the use of knowledge distillation, reinforcement learning, and other means make up for the loss of accuracy caused by optimizing convolution.

## Figures and Tables

**Figure 1:** Data set format: (a–c) chest radiograph medical images of ordinary pneumonia, and (d–f) chest radiograph medical images of confirmed pneumonia. It can be roughly seen from the figure that the chest texture structure of the routine chest radiograph is more straightforward than that of the pneumonia chest radiograph.

**Figure 2:** ResNet50 structure before and after pruning. The left side of the figure is a schematic diagram of the beginning of the original ResNet50 and the structure of the first two bottleneck blocks. The right side is the structure of CPResNet50 after pruning, which represents the pruning rate of the first convolutional layer. Each bottleneck block contains three convolutional layers; a normalization layer follows each convolutional layer. Finally, an activation function introduces nonlinear factors for channel transmission (one more convolutional layer and normalization layer at the Bottleneck).

The article "Auxiliary Pneumonia Classification Algorithm Based on Pruning Compression" was published in 2022. Journal: Comput Math Methods Med.

**Figure 3:** Channel pruning structure diagram in the figure; *X* is the output of the upper convolution, and then in the convolution layer, the weight of the BN layer is used to perform a simple sorting operation from small to large, and then the pruning rate *λ*_*i*_ of this layer is used to BN-weight. Pruning is performed from small to large, and the remaining feature maps are used as the input of the lower convolutional layer, and the pruning operation is continued in the *i* + 1 layer.

**Figure 4:** The convolution decomposition structure diagram: the gray part in the figure is the pruned feature map, the dark green part in the middle part is the feature map obtained by standard convolution, and the light green unequal is the “cheap feature map” generated by a linear transformation, and *Φ*_*i*_ denotes the cheap operation of the convolution of this layer.

**Figure 5:** ResNet50 channel pruning structure. (a) The structure of the original ResNet50; (b) the fusion work part of channel pruning and optimized convolution.

**Figure 6:** On ResNet50, the accuracy, and Flops line graph of CPG, SP, and CP methods, the left side is the accuracy graph line graph, and the right side is the Flops line graph.

**Table 1:** Comparison of different pruning rates between SR and CP methods on ResNet50.

Model	Test acc (%)	Parameters (M)	Pruned (%)	FLOPs (GFlops)	Pruned (%)
ResNet50 (normal)	97.827	23.512	—	4.12	—
SResNet50 (10% pruned)	97.707	21.58	10	3.43	8.22
SResNet50 (30% pruned)	98.129	17.222	30	2.64	26.75
SResNet50 (50% pruned)	97.526	12.278	50	1.85	47.78
SResNet50 (70% pruned)	97.888	7.466	70	1.21	68.25
CPResNet50 (10% pruned)	97.586	20.359	10	3.43	13.41
CPResNet50 (30% pruned)	97.707	14.942	30	2.43	36.45
CPResNet50 (50% pruned)	98.189	10.337	50	1.70	56.04
CPResNet50 (70% pruned)	97.707	6.682	70	1.15	71.58
CPResNet50 (80% pruned)	98.129	5.16	80	0.94	78.05
CPResNet50 (90% pruned)	97.888	3.888	90	0.696	83.46

**Table 2:** Comparison of CP method with other network models at different pruning rates.

Model	Test acc (%)	Params (M)	MAdd (G)	FLOPs (G)
CPResNet50 (50% pruned)	98.189	10.337	3.68	1.85
CPResNet50 (70% pruned)	97.707	6.682	2.4	1.21
CPResNet50 (90% pruned)	97.888	3.888	1.38	0.696
VGG16 [36]	96.619	14.773	30.77	15.41
DenseNet121 [37]	97.948	6.956	5.74	2.88
GoogLeNet [38]	98.371	5.60	3.02	3.02
Inception_v3 [39]	93.784	21.79	5.69	2.85

The article "Auxiliary Pneumonia Classification Algorithm Based on Pruning Compression" was published in 2022. Journal: Comput Math Methods Med.

**Table 3:** Comparison of different pruning rates between CP and CPG methods on ResNet50.

Model	Test acc (%)	Parameters (M)	Pruned (%)	FLOPs (G)	Pruned (G)
ResNet50 (normal)	97.827	23.512	—	4.12	—
GResNet50	98.430	13.317	—	2.32	43.36
CPResNet50 (10% pruned)	97.586	20.359	10	3.55	13.41
CPGResNet50 (10% pruned)	96.922	11.734	10	2.04	50.09
CPResNet50 (30% pruned)	97.707	14.942	30	2.64	36.45
CPGResNet50 (30% pruned)	97.224	10.336	30	1. 85	61.66
CPResNet50 (50% pruned)	98.189	10.337	50	1.85	56.04
CPGResNet50 (50% pruned)	97.043	9.015	50	1. 58	56.04
CPResNet50 (70% pruned)	97.707	6.682	70	1.21	71.58
CPGResNet50 (70% pruned)	96.922	4.863	70	1.18	79.32
CPResNet50 (80% pruned)	98.129	5.16	80	0.94	78.05
CPGResNet50 (80% pruned)	97.103	4.096	80	0.715	82.58
CPResNet50 (90% pruned)	97.888	3.888	90	0.696	83.46
CPGResNet50 (90% pruned)	97.745	3.455	90	0.591	85.31

**Table 4:** Comparison of CPGResNet50 (90% pruned) and lightweight model.

Model	Test acc (%)	Parameters	FLOPs
MobileNetV2 [21]	97.069	2.226 M	318.96 M
ShuffleNetV2 [24]	97.431	0.344 M	42.62 M
CPGResNet50 (90% pruned)	97.75	3.455 M	591 M

## Data Availability

Data is available on request from the authors due to privacy/ethical restrictions.
